# Evaluation of Neutrophil-Lymphocyte Ratio and Platelet-Lymphocyte Ratio on Predicting Responsiveness to Neoadjuvant Chemoradiotherapy in Locally Advanced Rectal Cancer Patients

This article has been retracted.

**DOI:** 10.1155/2022/3839670

**Published:** 2022-09-28

**Authors:** Maoxi Liu, Yi Feng, Yixun Zhang, Haiyi Liu

**Affiliations:** Department of Anorectal Surgery, Shanxi Cancer Hospital, Taiyuan, 030013 Shanxi, China

## Abstract

**Objective:**

Neutrophil-lymphocyte ratio (NLR) and Platelet-lymphocyte ratio (PLR) have been proposed as prognostic biomarkers in multiple cancers. However, the implications of NLR and PLR in the responsiveness to neoadjuvant chemoradiotherapy (nCRT) remain to be clarified in locally advanced rectal cancer (LARC) patients. This retrospective study investigated the prognostic value of NLR and PLR in nCRT responsiveness of LARC patients.

**Methods:**

A total number of 86 patients diagnosed with LARC and treated with nCRT and total mesorectal excision were retrospectively followed from 2013 to 2016. Receiver operating characteristic (ROC) curve was used to determine the cutoff values of NLR and PLR, and the patients were divided into NLR elevation and NLR decrease groups, or PLR elevation and PLR decrease groups. The correlation between NLR and PLR changes, and clinicopathological factors were analyzed. The relationship between NLR and PLR changes and the curative responsiveness towards nCRT were further evaluated.

**Results:**

NLR and PLR changes after nCRT were significantly correlated with the distance of tumors to the anus and BMI (body mass index) (*P* < 0.05). The clinical remission rate of patients with NLR reduction was 72.09% (31/43), which was significantly higher than that in patients with NLR increment (22/43, 51.16%). There was no significant difference in the clinic remission rate between the patients with PLR reduction and those with PLR increment (*P* > 0.05). However, the pathological responsiveness rate was significantly higher in patients with PLR reduction (21/43, 48.84%) when compared to the ones with PLR increment (9/43, 20.9%) (*P* = 0.036).

**Conclusion:**

Our data indicate that in LARC patients with nCRT, the reduction of NLR and the reduction of PLR could serves as predictors for the clinic remission rate and pathological responsiveness rate, respectively. The combination of NLR and PLR changes may be employed as a simple and effective prognostic parameter to predict the treatment outcome of nCRT in LARC.

## 1. Introduction

Colorectal cancer remains as one of the most commonly diagnosed solid tumors and the leading cause of cancer-related lethality worldwide [1]. Despite the advancement of the diagnostic and therapeutic approaches, patients with colorectal cancer suffer from a poor over survival (OS), with fewer than 20% surviving beyond 5 years from diagnosis. Furthermore, about 25% rectal cancer patients are diagnosed at locally advanced stage with tissue invasion, which restricts the efficacy of the optimal surgical resection. Fluoropyrimidine-based concurrent neoadjuvant chemoradiotherapy (nCRT) followed by total mesorectal excision (TME) is the mainstay of the standard-of-care treatment in LARC patients [2]. Nevertheless, different patients show distinct responsiveness to nCRT. Patients who respond to nCRT with conclusive evidence in radiography and pathology have been shown to have improved long-term outcomes, such as disease-free survival (DFS) and over survival (OS) [3, 4]. Therefore, the stratification of patients by predicting the responsiveness to nCRT is of clinical significance for the selection of the optimal treatment strategy. Ren et al. reported that about 8%-35% LARC patient after nCRT could achieve a complete pathological response, and no surgery was further required [5]. However, currently there are no effective predictors to judge the efficacy of nCRT in LARC patients.

Chronic inflammation has been recognized as a contributing factor facilitating cancer initiation and progression [6]. Accumulating evidence suggests that systemic inflammatory response is a hallmark of malignant progression in cancers which is associated with the poor outcome of cancer patients [6, 7]. Neutrophils, lymphocytes, and platelets are key players in systemic inflammatory response [8]. Neutrophil-lymphocyte ratio (NLR) is defined as the absolute neutrophil count divided by the absolute lymphocyte count, and platelet-lymphocyte ratio (PLR) is defined as the absolute platelet count divided by the absolute lymphocyte count. NLR and PLR have been suggested as potential prognostic biomarker in multiple cancers [9]. The correlations between immunologic biomarkers including NLR and PLR and the prognosis in colorectal cancer patients have also been reported [10–15]. However, there seem to be conflicting results that whether NLR and PLR can serve as effective prognostic predictor in rectal cancer [12, 16]. In addition, the potential implications of NLR and PLR in nCRT responsiveness remain to be clarified. In this retrospective study, we investigated the prognostic value of NLR and PLR in nCRT responsiveness of LARC patients.

## 2. Materials and Methods

### 2.1. Patient Sample

Data were analyzed from a total of 86 patients diagnosed with LARC and treated with nCRT followed by TME. The inclusion criteria are the following: the diagnosis of LARC in all patients were histologically verified by experienced pathologists; all the patients had an American Society of Anesthesiologist Physical Status Classification score lower than 2; CT scan of the chest and upper abdomen indicated no distant metastasis; pelvic MR (magnetic resonance) suggested that rectal cancer was in locally advanced stage; all patients were treated nCRT, with consisted of two-three cycles of chemotherapy (consisting of capecitabine at the dose of 2500 mg/m^2^ for two weeks, with one recovery week; oxaliplatin at the dose of 85 mg/m^2^ combined with capecitabine at the dose of 2500 mg/m^2^ or fluorouracil at the dose of 2800/m^2^ every two weeks) and pelvic radiotherapy (RT) (RT was performed as conventional fractionation using 6-10 MV photo beams and was delivered at a dose of 1.8-2.0 Gy to a total dose of 50 Gy over 4 weeks); electronic medical records of the clinicopathological parameters such as sage, gender, BMI, histology, performance stage, clinical stage, RT dose, chemotherapy, and blood cell count were complete; all patients had not been diagnosed with other cancers before. This study was approved by the Medical Ethics Committee of the Shanxi Cancer hospital on 24 March, 2013.

Laparoscopic radical resection was performed for LARC patients. The operation follows the criteria of total mesorectal excision (TME) and lymph node dissection. The operation mainly includes laparoscopic exploration, free sigmoid colon and rectum through medial approach, high ligation of submesenteric vessels, and dissection of lymph nodes, removal of specimens and reconstruction of bowel. The pneumoperitoneum (14 mmHg) (1 mmHg = 0.133 kPa) was established by the five hole method. The peritoneum was incised in the anterior direction of the sacral promontory. After the root of the inferior mesenteric artery was dissected, the inferior mesenteric vein was clamped at a distance of 1 cm from the root. The inferior mesenteric vein was treated in the same manner to free the colon mesentery from the inside to the outside, sharply separate the space between the fascia of the basin wall and the fascia proper to the rectum, and then from the posterior part of the rectum to the plane of the tip of the tailbone. After completing the above operations, the specimen was taken out, and the intestinal reconstruction was performed. According to the consensus of experts on the diagnosis, prevention and treatment of anastomotic leakage in rectal cancer surgery in China, whether to make a stoma was decided.

### 2.2. Assessment of nCRT Responsiveness

#### 2.2.1. Clinical Curative Responsiveness Assessment

CT scan in the chest and upper abdomen and MR scan in the pelvic were used to assess the clinical curative responsiveness 6-8 weeks after nCRT. The efficacy of nCRT was evaluated by the guidelines of the Response Evaluation Criteria In Solid Tumors (RECIST) [17], which includes complete response (CR, all tumor lesions disappeared, no new lesions appeared), partial response (PR, the sum of the maximum diameters of tumor lesions decreased by ≥30%), stable (SD, the sum of the maximum diameters of the tumor lesions was unreachable to PR and unreachable to PD), and progression (PD, the sum of the maximum diameters of tumor lesions increased by ≥20%). The response rate is calculated as (CR + PR)/(CR + PR + SD + PD) × 100%.

#### 2.2.2. Pathological Responsiveness Categorization

After nCRT therapy, the sections of surgical tumor tissues were subjected to hematoxylin-eosin (HE) staining for pathological responsiveness categorization. The Miller-Payne criteria were used to grade pathological responsiveness of solid tumor to nCRT as follows [18]:

*Grade 1*. No change or only minor change in malignant cells, and no reduction in total cellularity.

*Grade 2*. Minor loss of tumor cells with up to 30% reduction in cellularity.

*Grade 3*. 30%-90% reduction of tumor cells.

*Grade 4*. >90% reduction of tumor cells and only small clusters of dispersed tumor cells remained.

*Grade 5*. No invasive malignant cells identifiable.

Patients with grade 1 to 3 diagnoses were classified as nCRT nonresponsive group, and patients with Grade 4 and 5 diagnoses were considered as nCRT responsive group. The workflow of the study is shown in Figure 1.

### 2.3. Determine the Optimal Cutoff Values

The optimal cutoff values for PLR and NLR to predict effective of NCRT were identified by receiver operating characteristic (ROC) curve.

### 2.4. Statistical Analysis

SPSS 21.0 software package was used for statistical analysis. All continuous variables were expressed as mean ± standard deviation (SD). Student's *t* or *χ*2 test was used to calculate the statistical differences between groups. In all analyses, *P* < 0.05 was considered as statistically significant.

## 3. Results

### 3.1. Correlation of Clinicopathological Parameters with the Change of NLR and PLR after nCRT

The data from 86 patients with the diagnosis of LARC and treated with nCRT between March 2013 and September 2016 were analyzed. The median age of LARC patients was 60 years (range, 38-72 years) with 57 males (66.3%) (Table 1). The physical performance of the patients was satisfactory after nCRT. (Eastern Cooperative Oncology Group, ECOG value ≤ 1). The percentage of patients with tumor distance to anus less than 6 cm was 41.9%, and percentages of patients diagnosed with TNM (tumor node metastasis classification) Stage II and Stage III were 36 (41.9%) and 50 (58.1%), respectively (Table 1).

Based on the median fraction of the NLR and PLR changes pre- and postnCRT, eight-six patients were divided into elevation group and decrease group of the changes. There were 43 cases in the NLR elevation group and decrease group, respectively. Between the two groups, there were no significant changes between age, gender, TNM stage, lymph node of metastasis, and tumor diameters (Table 2, P > 0.05). However, the NLR decrease group was associated with more cases of tumor distance to anus ≥ 6 cm and more cases of BMI < 28 after nCRT (Table 2, *P* < 0.05). In terms of PLR change, PLR decrease group was also significantly associated with more cases of tumor distance to anus ≥ 6 cm and more cases of BMI < 28 after nCRT (Table 3, *P* < 0.05).

### 3.2. Correlation between the Changes in NLR and PLR and Curative Responsiveness before and after nCRT

To optimize the cutoff values for PLR and NLR after nCRT to predict effectiveness of prenCRT, the receiver operating characteristic (ROC) curve analysis was performed. The cutoff values were 2.3 for NLR and 142.44 for PLR. In addition, the area under the curve (AUC) for PLR and NLR was 0.657 (*P* = 0.051, 95% CI: 0.531-0.750) and 0.648 (*P* = 0.553, 95% CI: 0.442-0.665), respectively. The optimal cutoff values postnCRT were 2.05 for NLR and 152.75 for PLR. Besides, the AUC for PLR and NLR was 0.619 (*P* = 0.224, 95% CI: 0.512-0.716) and 0.649 (*P* = 0.145, 95% CI: 0.513-0.723), respectively (Figure S1). As shown in Table 4, the response rate was 72.09% (31/43) in NLR decrease group and was 51.16% (31/43) in NLR elevation group. Importantly, there was a significant increase in the responsive cases in NLR decrease group in comparison to the NLR elevation group (*χ*^2^ = 3.983, *P* = 0.046). However, there was no significant difference in the curative responsiveness between PLR decrease and PLR elevation groups (*χ*^2^ = 1.229, *P* = 0.268).

### 3.3. Correlation between NLR and PLR Changes and the Pathological Responsiveness before and after nCRT

As shown in Table 5, the pathological response was 48.84% (21/43) in PLR decrease group and was 20.93% (9/43) in PLR elevation group, and there was a significant increase in the responsive cases in PLR decrease group in comparison to the PLR elevation group (*χ*^2^ = 4.472, *P* = 0.036). However, there was no significant difference in the pathological responsiveness between NLR decrease and NLR elevation groups (*χ*^2^ = 0.199, *P* = 0.655).

## 4. Discussion

Inflammation has been recognized as a key factor in cancer microenvironment that contributes to the occurrence and progression of multiple tumors. As the marker of inflammation, the clinical implications of NLR and PLR in the prognosis of cancer patients have been widely studied in various tumors [9]. Recent works have demonstrated that NLR and PLR are not only associated with poor prognosis but also have diagnostic value in colorectal cancer [18, 19]. In this study, we investigated the relationship between NLR and PLR changes and nCRT responsiveness in LARC patients. Our data showed that the changes of NLR and PLR before and after nCRT were significantly associated with BMI, which seemed to be consistent with a previous report by Li et al. [19]. We also found that the changes of NLR and PLR were significantly associated with the distance of tumor to anus, indicating the correlation between the localization of tumor in the colon and difference in the activity of different immune components.

Several studies suggested that the elevation of perioperative NLR is a prognostic factor for worse outcome in LARC patients, while the decrease of NLR suggests a better prognosis [11, 14]. However, some studies showed an opposite trend of the relationship between NLR change and the overall survival [12, 16]. Our data demonstrated that the clinical remission rate of LARC patients with NLR reduction was 72.09% (31/43), which was significantly higher than NLR elevation group (51.16%). This result suggests that NLR reduction after nCRT indicates a good curative effect, which is consistent with a previous report by Ya et al. [20]. A possible explanation is that neutrophils promote tumor growth by inactivating lymphocyte and T-cell response [21, 22]. nCRT combined with immune-potentiator has been shown to boost immune function during cancer treatment [23]. In addition, nCRT can also impact on the tumor microenvironment, and neutrophils can promote angiogenesis through producing vascular endothelial growth factor [24].

PLR is another commonly investigated inflammatory index, which has been shown to be associated with tumor proliferation and angiogenesis [25, 26]. Activated platelet secretes a number of growth factors such as platelet-derived growth factor (PDGF), which can support the malignant progression of cancer [25, 26]. High PLR was reported to be associated with poor prognosis in LARC patients [27]. In our study, we also found that the pathological response in patients with PLR reduction was 48.84% (21/43), which was significantly higher than that of PLR elevated group (20.93%). Our results are consistent with the findings by Lee et al. [28]. Together, these results suggest that PLR change after nCRT in LARC patients is an important predictor of pathological response.

Our study suffers from some limitations. First, this study was single-central and retrospective study, and there may be a selection bias of the participants enrolled. A prospective multicenter randomized study could provide the validation of current findings. In addition, the enrolled cohort is small and the external validation with a larger cohort of LARC patients can provide more convincing conclusions. It is worth mentioning that neither NLR nor PLR alone can provide sufficient prediction of the response to nCRT. Therefore, the combination of NLR and PLR changes may serve as a better predictor for the responsiveness of LARC patients towards nCRT.

## 5. Conclusions

In summary, we reported that the changes of NLR and PLR pre- and postnCRT were significantly associated with the clinical responsiveness towards nCRT. The clinical remission rate of patients with NLR reduction was significantly higher than that in patients with NLR increase, while the pathological responsiveness rate was significantly higher in patients with PLR reduction. Our data imply that the combination of NLR and PLR changes may be employed as a better index for predicting the clinical responsiveness of LARC patients towards nCRT.

## Figures and Tables

**Figure 1:** Schematic workflow of the study involving LARC patients and NRL/PLP analysis before and after nCRT treatment.and

**Table 1:** Patient clinicopathological parameters.

Characteristics	*n* (%)
Age (years)	
> 60	17 (18.8)
≤ 60	69 (81.2)
Gender	
Male	57 (66.3)
Female	29 (33.7)
Distance to anus (cm)	
≥ 6	36 (41.9)
< 6	50 (58.1)
BMI (kg/m^2^)	
≥ 28	11 (12.8)
< 28	75 (87.2)
TNM	
II	36 (41.9)
III	50 (58.1)
Number of lymph node metastasis and nodules	
> 3	19 (22.1)
≤ 3	67 (77.9)
Diameter of tumor	
> 3	38 (44.2)
≤ 3	48 (55.8)

**Table 2:** Relationship between NLR change and clinicopathological factors after nCRT.

Characteristics	Cases	NLR elevated	NLR decreased	*χ*2	*P*
Age (years)				0.660	0.417
> 60	17	7	10		
≤ 60	69	36	33		
Gender				0.052	0.820
Male	57	28	29		
Female	29	15	14		
Distance to anus (cm)∗				4.778	0.029
≥ 6	36	13	23		
< 6	50	30	20		
TNM stage				0.764	0.382
III	50	23	27		
II	36	20	16		
BMI (kg/m^2^)				5.108	0.024
≥ 28	11	9	2		
< 28	75	34	41		
Lymph node of metastasis and nodules				3.310	0.069
> 3	19	6	13		
≤ 3	67	37	30		
Diameter of tumor (cm)				0.754	0.385
> 3	38	17	21		
≤ 3	48	26	22		

^∗^Distance to anus (cm): the distance between the lower edge of the tumor and the anal edge.

**Table 3:** Relationship between PLR change and clinicopathological factors after nCRT.

Characteristics	Cases	PLR elevated	PLR decreased	*χ*2	*P*
Age (years)				0.660	0.417
> 60	17	10	7		
≤ 60	69	33	36		
Gender				0.468	0.494
Male	57	30	27		
Female	29	13	16		
Distance to anus (cm)				9.364	0.002
≥ 6	36	11	25		
< 6	50	32	18		
TNM stage				1.720	0.190
III	50	22	28		
II	36	21	15		
BMI (kg/m^2^)				8.444	0.004
≥ 28	11	10	1		
< 28	75	33	42		
Lymph node of metastasis and nodules				1.689	0.194
> 3	19	7	12		
≤ 3	67	36	31		
Diameter of tumor (cm)				0.754	0.385
> 3	38	17	21		
≤ 3	48	26	22		

**Table 4:** Relationship between changes in NLR and PLR and curative responsiveness before and after nCRT.

Groups	Cases	Responsive (CR + PR)	Nonresponsive (SD + PD)	*χ*2	*P*
NLR (pretreatment)				0.049	0.825
> 2.30	43	26 (60.47)	17 (39.53)		
≤ 2.30	43	27 (62.79)	16 (37.21)		
PLR (pretreatment)				0.049	0.825
> 142.44	43	26 (60.47)	17 (39.53)		
≤ 142.44	43	27 (62.79)	16 (37.21)		
NLR (posttreatment)				2.409	0.121
> 2.05	43	23 (53.49)	20 (46.51)		
≤ 2.05	43	30 (69.77)	13 (30.23)		
PLR (posttreatment)				2.409	0.121
> 152.75	43	23 (53.49)	20 (46.51)		
≤ 152.75	43	30 (69.77)	13 (30.23)		
NLR change				3.983	0.046
Elevated group	43	22 (51.16)	21 (48.84)		
Decreased group	43	31 (72.09)	12 (27.91)		
PLR change				1.229	0.268
Elevated group	43	24 (55.81)	19 (44.19)		
Decreased group	43	29 (67.44)	14 (32.56)		

**Table 5:** Relationship between NLR and PLR changes and the pathological responsiveness before and after nCRT.

Groups	Cases	Pathologically responsive	Pathologically nonresponsive	*χ*2	*P*
NLR (pretreatment)					
> 2.30	43	18 (41.86)	25 (58.14)	0.048	0.826
≤ 2.30	43	17 (39.53)	26 (60.47)		
PLR (pretreatment)					
> 142.44	43	15 (34.88)	28 (65.12)	0.050	0.822
≤ 142.44	43	16 (37.21)	27 (62.79)		
NLR (posttreatment)					
> 2.05	43	16 (37.21)	27 (62.79)	0.434	0.510
≤ 2.05	43	19 (44.19)	24 (55.81)		
PLR (posttreatment)					
> 152.75	43	18 (41.86)	25 (58.14)	0.094	0.759
≤ 152.75	43	17 (39.53)	27 (61.47)		
NLR change					
Elevated group	43	17 (39.53)	26 (61.47)	0.199	0.655
Decreased group	43	15 (34.88)	28 (65.12)		
PLR change					
Elevated group	43	9 (20.93)	34 (79.07)	4.472	0.036
Decreased group	43	21 (48.84)	22 (51.16)		

## Data Availability

All data generated or analyzed during this study are included in this paper. Further enquiries can be directed to the corresponding author.

## Supplementary Materials

Supplementary Materials Figure S1. Receiver operating characteristic (ROC) curve analysis of PLR and NLR in both prenCRT and postnCRT LARC patients. AUC: area under the curve; CI: confidence interval.
